This article has been retracted.

# BRMS1 Suppresses Glioma Progression by Regulating Invasion, Migration and Adhesion of Glioma Cells

**DOI:** 10.1371/journal.pone.0098544

**Published:** 2014-05-30

**Authors:** Pengjin Mei, Jin Bai, Meilin Shi, Qinghua Liu, Zhonglin Li, Yuechao Fan, Junnian Zheng

**Affiliations:** 1 Department of Neurosurgery, The Affiliated Hospital of Xuzhou Medical College, Xuzhou, Jiangsu, China; 2 Jiangsu Key Laboratory of Biological Cancer Therapy, Xuzhou Medical College, Xuzhou, Jiangsu, China; 3 Department of Medical Oncology, The Affiliated Hospital of Xuzhou Medical College, Xuzhou, Jiangsu, China; Aix-Marseille University, France

## Abstract

Breast cancer metastasis suppressor 1 (BRMS1) is a metastasis suppressor gene in several solid tumors. However, the expression and function of BRMS1 in glioma have not been reported. In this study, we investigated whether BRMS1 play a role in glioma pathogenesis. Using the tissue microarray technology, we found that BRMS1 expression is significantly decreased in glioma compared with tumor adjacent normal brain tissue (*P*<0.01, χ^2^ test) and reduced BRMS1 staining is associated with WHO stages (*P*<0.05, χ^2^ test). We also found that BRMS1 was significantly downregulated in glioma cell lines compared to normal human astrocytes (*P*<0.01, χ^2^ test). Furthermore, we demonstrated that BRMS1 overexpression inhibited glioma cell invasion by suppressing uPA, NF-κB, MMP-2 expression and MMP-2 enzyme activity. Moreover, our data showed that overexpression of BRMS1 inhibited glioma cell migration and adhesion capacity compared with the control group through the Src-FAK pathway. Taken together, this study suggested that BRMS1 has a role in glioma development and progression by regulating invasion, migration and adhesion activities of cancer cells.

## Introduction

Gliomas are the most common primary malignancies in the central nervous system (CNS). According to the World Health Organization (WHO) [1], gliomas are classified into four grades as follows: pilocytic astrocytoma, WHO grade I; diffuse “low grades” glioma, WHO grade II; anaplastic gliomas, WHO grade III; and glioblastoma (GBM), WHO grade IV. GBM, is one of the most aggressive and lethal forms of cancer with an average survival time of 15 months after diagnosis [2]. Invasion is usually recognized as the main reason for the high recurrence and death rates of glioma and migration of tumor cells plays an important role in the invasion of glioma and restricts the efficacy of surgery and other therapies [3]. Therefore, understanding the molecular mechanisms of glioma invasion and migration is an urgent challenge in the development of new therapeutic strategies for this deadly disease.

Breast cancer metastasis suppressor 1 (BRMS1) was identified by differential display comparing metastasis-suppressed chromosome 11 hybrids with metastatic, parental MDA-MB-435 human breast carcinoma cells [4], and BRMS1 has subsequently been shown to suppress metastasis, but not tumorigenicity, of human melanoma and ovarian cancer cells in nude mice [5], [6]. Recent studies have indicated that BRMS1 expression was reduced in breast cancer, melanoma, ovarian cancer, nasopharyngeal carcinoma and non-small cell lung cancer (NSCLC), and seemed to be associated with cancer cell invasion, metastasis and patients' prognosis [6]–[12]. There are several proposed mechanisms of action for BRMS1 and its role in the regulation of tumor metastasis; these include restoration of gap junctions, reduction of phosphoinositide signaling, interaction with the histone deacetylase complex and regulation of the nuclear factor-κB (NF-κB) pathway [13]–[15]. Specially, several metastasis-related genes were found to be downregulated by BRMS1 through modulating the activity of NF-κB, including osteopontin (OPN), urokinase-type plasminogen activator (uPA), micro-RNA-146, interleukin-6 (IL-6) and chemokine receptor 4 (CXCR4) [9], [16]–[20]. Until recently, limited data existed on the role of BRMS1 in glioma.

In this study, we used a tissue microarray (TMA) of human glioma patients and immunohistochemistry to evaluate the expression of BRMS1 in relation to clinicopathologic features. We found that BRMS1 expression was significantly decreased in glioma compared with tumor adjacent normal brain tissue and this reduced expression was associated with WHO stage. We report that BRMS1 was significantly downregulated in glioma cells compared to normal human astrocytes (NHA). We then demonstrated that BRMS1 overexpression suppressed glioma cell invasion, migration and adhesion abilities. In addition, we investigated the molecular mechanisms underlying BRMS1 actions in glioma cells.

## Materials and Methods

### Data availability statement

Data is available to researchers upon request.

### Ethics statement

This study was performed under a protocol approved by the Institutional Review Boards of The Affiliated Hospital of Xuzhou Medical College and all examinations were performed after obtaining written informed consents.

### Patients and samples

A glioma TMA was purchased from Shanxi Alenabio Biotechnology (xi'an, China), No: GL2083a. Pathologic grades of tumors were defined according to the 2000 WHO criteria as follows: 134 cases of benign tumor (Grade I and II), 58 cases of malignant tumor (Grade III and IV), 8 cases of tumor adjacent normal brain tissue and 8 cases of normal brain tissue. The array dot diameter was 1.0 mm, and each dot represented a tissue spot from one individual specimen that was selected and pathologically confirmed. Four paired glioma tissues and adjacent non-tumor tissues from the same patients were obtained from the Department of Neurosurgery, the affiliated hospital of Xuzhou Medical College.

### Immunohistochemistry of TMA

The TMA slides were dewaxed by heating at 55°C for 30 min and by three washes, 5 min each, with xylene. Tissues were rehydrated by a series of 5 min washes in 100, 95, and 80% ethanol and distilled water. Antigen retrieval was performed by heating the samples at 95°C for 30 min in 250 ml of 10 mmol/L sodium citrate (pH 6.0). Endogenous peroxidase activity was blocked with 0.3% hydrogen peroxide for 20 min. Nonspecific binding was blocked with goat serum for 30 min. The primary monoclonal rabbit anti-BRMS1 antibody (Abcam, Cambridge, MA) was diluted 1∶400 using goat serum and incubated at room temperature for 1 hour. After three washes, 2 min each with PBS, the sections were incubated with a biotinylated goat anti-rabbit secondary antibody for 30 min (Zhongshan Biotech, Beijing, China), followed by the incubation with streptavidin-peroxidase (Zhongshan Biotech, Beijing, China) for an additional 30 min. After rinsing with PBS 3 times for 2 min, the sections were stained using DAB (Zhongshan Biotech, Beijing, China) for 15 min, rinsed in distilled water and counterstained with hematoxylin. Dehydration was then performed following a standard procedure, and the sections were sealed with cover slips. Negative controls were performed by omitting BRMS1 antibody during the primary antibody incubation.

### Evaluation of immunostaining

The BRMS1 staining was examined double-blinded by two independent pathologists, and a consensus was reached for each core. The expression of BRMS1 was graded as positive when over 5% of tumor cells showed immunopositivity. Biopsies with less than 5% tumor cells showing immunostaining were considered as negative [21].

### Cell culture and transfection

Primary normal human astrocytes (NHA) were purchased from the KeyGEN Biotech Company (Nanjing, China) and cultured under the conditions as instructed by the manufacturer. Human glioma cell lines (U251, U87, T98G, SHG44) and Rat glioma cell C6 were purchased from the Institute of Biochemistry and Cell Biology, Chinese Academy of Science. All glioma cells were cultured in DMEM supplemented with 10% fetal bovine serum (Invitrogen, Shanghai, China) at 37°C in 5% CO_2_.

The pFlag-control and pFlag-BRMS1 expression plasmids were a gift from Dr Shouyi Qiao (Fudan University, China). Transfection of the pFlag-control and pFlag-BRMS1 plasmids into the U251 and U87 glioma cells were carried out using Lipofectamine 2000 transfection reagent (Invitrogen, Shanghai, China) following the manufacturer's instructions. 6 hours after transfection, the medium containing transfection reagents was removed. The cells were rinsed twice with PBS and incubated in fresh medium. 24 hours after transfection, cells were lysed for Western blot assay, and cell proliferation assay, cell matrigel invasion assay, migration assay and adhesion assay.

To measure the transfection efficiency, we transfected the GFP plasmid into the U251 and U87 glioma cells and used fluorescence-activated cell sorting (FACS) to detect the efficiencies of U251 and U87 cells. The efficiencies of U251 and U87 were 90.8% and 83.1%, respectively.

### Western blot analysis

Cells were harvested and washed thrice with PBS. Whole cell proteins were extracted as described previously [22]. Protein concentrations were determined by protein assay (Bio-Rad, Hercules, CA, USA). Western blot analysis was done as described previously [23]. The following antibodies were used for Western blot: rabbit anti-BRMS1 (Abcam, Cambridge, MA), rabbit anti-FAK, Src, MMP-2, uPA, NF-κB (all from Cell Signaling Technology, Beverly, MA, USA) and mouse anti-β-actin (Zhongshan Biotech, Beijing, China). Infrared IR dye-labeled secondary antibody was applied to the blot for 1 hour at room temperature. The signals were detected with Odyssey IR Imaging system (LI-COR, Lincoln, NE).

### Cell proliferation assay

Cell proliferation was analyzed using a WST-8 Cell Counting Kit-8 (CCK-8) (Beyotime, Nantong, China); 3×10^3^ cells suspended in 100 µl DMEM medium containing 10% fetal bovine serum were seeded in 96-well plates and incubated for 24, 48, 72 and 96 hour; 10 µl CCK-8 solution was added to each well and the cultures were incubated at 37°C for 1 hour. Absorbance at 450 nm was measured on an ELX-800 spectrometer reader (Bio-Tek Instruments, Winooski, USA).

### Invasion assay

Cell invasion was assessed by matrigel precoated Transwell inserts (8.0 µm pore size with polyethylene tetraphthalate membrane) according to the manufacturer's protocol. To assess invasion, filters were precoated with 10 µg of matrigel (BD Biosciences, NJ, USA). 1×10^5^ cells were seeded in serum-free medium in the upper chamber. After 24 hour incubation at 37°C, cells in the upper chamber were carefully removed with a cotton swab and the cells that had traversed the membrane were fixed in methanol, stained with Giemsa. Five separate fields of cells on the underside of the filters were photographed and counted.

### Wound healing assay

After U251 and U87 glioma cells were transfected with the BRMS1 and control plasmids, cells were cultured in fresh medium for 24 hours and treated with 10 µg/ml mitomycin C for 2 hours. After washing with PBS, a standard 200 µl pipette tip was drawn across the center of each well to produce a wound of ∼0.5 mm in width. The wounded monolayers were washed twice to remove non-adherent cells, and fresh medium was added. The photos were taken at the same position of the wound at various time intervals. The starting wound edges were defined in each photo by white lines according to the scratch at 0 hour time point. The wound-healing percentage was determined by the ratio of healing width at each time point to the wound width at 0 h. Experiments were carried out in triplicate, and three random fields of each well were recorded.

### Migration assay

Cell migration was determined by using a modified two chamber migration assay with a pore size of 8 µm. For migration assay, 1×10^5^ cells were seeded in serum-free medium in the upper chamber. After 12 hour incubation at 37°C, cells in the upper chamber were carefully removed with a cotton swab and the cells that had traversed the membrane were fixed in methanol, stained with Giemsa. Five separate fields of cells on the underside of the filters were photographed and counted.

### Cell attachment assay

96-well plates were coated with 1.25 µg/ml fibronectin (BD Biosciences, NJ, USA) in 100 µl PBS overnight at 4°C. Wells coated with bovine serum albumin (BSA) served as negative control. The plates were blocked with 2.5 mg/ml BSA for 2 hour in DMEM at 37°C. Cells were trypsinized and 2×10^4^ cells were seeded in each well for 1 hour at 37°C, and then the cell adhesion assay was performed as previously described [24].

### Gelatin zymography

2×10^6^ cells were seeded in 100 mm plate for 24 hour, cells were transfected with the BRMS1 and control plasmids. 24 hours after transfection, serum-free medium was applied to the cells overnight and the proteins in the conditioned medium were concentrated with Ultracel-30k centrifugal filters (Millipore, Billerica, MA) at 5,000×*g* for 20 min at 4°C. Proteins (50 µg) were loaded on a 10% polyacrylamide gel containing 0.1% gelatin (Sigma). After electrophoresis, gel was incubated in Triton X-100 exchange buffer (20 mM Tris-HCl [pH 8.0], 150 mM NaCl, 5 mM CaCl_2_ and 2.5% Triton X-100) for 30 min followed by 10 min wash with incubation buffer (same buffer without Triton X-100) thrice. The gel was then incubated in incubation buffer overnight at 37°C, stained with 0.5% Coomassie blue R250 (Sigma) for 4 hour and destained with 30% methanol and 10% glacial acetic acid for 2 hour. Gelatinolytic activity was shown as clear areas in the gel.

### Statistical analysis

Statistical analysis was performed with SPSS 16.0 software (SPSS, Chicago, IL). Data are expressed as the means ± SD. The association between BRMS1 staining and the clinicopathologic parameters of the glioma patients, including age, gender, WHO grade and histologic type, was evaluated by χ^2^ test. For CCK-8 cell proliferation assays, Student's *t* test was used. For the invasion assay, wound healing assay, migration assay and adhesion assay, the results were first quantified from three independent experiments and expressed as the means ± SD. And then the data were normalized to the control population. Differences were considered significant when *P*<0.05.

## Results

### BRMS1 expression is downregulated in glioma tissues and glioma cell lines

In order to investigate whether BRMS1 expression is changed in glioma, we utilized a TMA to evaluate the BRMS1 expression in normal brain tissue, tumor adjacent normal brain tissue, benign tumor (Grade I and II) and malignant (Grade III and IV). The representative pictures presented in Fig. 1A–D showed that BRMS1 protein mainly localized in cytoplasm was stained in brown. BRMS1 positive staining was observed in 5 of 8 (62.5%) normal brain tissue, 4 of 8 (50%) tumor adjacent normal brain tissue, 48 of 192 (25%) glioma tissue (Fig. 1E). A significant difference in BRMS1 staining was observed between normal brain tissue and glioma tissue (*P*<0.01, χ^2^ test) and between tumor adjacent normal brain tissue and glioma tissue (*P*<0.01, χ^2^ test). To further confirm these observations, Western blot assay was done using four glioma tissues and paired non-tumor tissues. It was clear that the glioma tissue had a drastic decrease of BRMS1 expression as compared with the non-tumor tissues (Fig. 1F), which was consistent with the level of BRMS1 protein expression determined by immunohistochemical staining. In addition, Western blot analyses showed that expression of BRMS1 was markedly lower in all 5 analyzed glioma cell lines, including SHG44, C6, U251, T98G, U87, as compared with that in normal human astrocytes (NHA) (Fig. 1G). Collectively, our results suggest that BRMS1 is downregulated in gliomas.

**Figure 1:** Representative images show BRMS1 immunohistochemical staining. **A** Positive BRMS1 staining in normal brain tissue (NB); **B** Positive BRMS1 staining in adjacent normal brain tissue (AB); **C** Negative BRMS1 staining in benign tumor (BT); **D** Negative BRMS1 staining in malignant tumor (MT); **E** A significant difference in BRMS1 staining was observed between normal brain tissue and glioma tissue (GT) (*P*<0.01, χ^2^ test) and between tumor adjacent normal brain tissue and glioma tumor (*P*<0.01, χ^2^ test). **F** Whole-cell protein extracts were further prepared from four paired tumor adjacent normal glioma tissues and glioma tissues. The BRMS1 protein level was determined by Western blot analysis. **G** Western blot analysis of BRMS1 expression in normal human astrocytes NHA and glioma cell lines, including SHG44, C6, U251, T98G, U87. **H** BRMS1 staining was dramatically decreased in malignant tumor compared with benign tumor (*P*<0.05). All experiments were carried out in triplicate. Data are shown as mean ± SD. *P<0.05, **P<0.01, ***P<0.001. Original magnification (**A–D**) ×40.

### BRMS1 expression is correlated with clinicopathological parameters

The clinicopathologic features of 192 glioma biopsies were summarized in Table 1. WHO grade and histologic type are known to be important prognostic markers for patients with glioma. We studied whether BRMS1 expression correlates with these markers. We found BRMS1 positive staining in 39 of 134 (29.1%) benign tumor and 9 of 58 (15.5%) malignant tumor. Therefore, BRMS1 staining was dramatically decreased in WHO stages III–IV compared with stages I–II (*P*<0.05, χ^2^ test, Fig 1H). However, we did not find significant correlations between BRMS1 expression and histologic type (Table 1). There is also no significant correlations between BRMS1 expression with other clinicopathologic variables, including patient age and gender (Table 1).

**Table 1:** BRMS1staining and clinicopathological characteristics of 192 glioma patients.

Variables	BRMS1 staining			
	Negative, No. (%)	Positive, No. (%)	Total	*P* *
**Age**				
<46 years	71(79.8%)	18(20.2%)	89	0.260
≥46 years	75(72.8%)	28(27.2%)	103	
**Gender**				
Male	90(76.9%)	27(23.1%)	117	0.721
Female	56(74.7%)	19(25.3%)	75	
**WHO Grade**				
Benign(I–II)	95(70.9%)	39(29.1%)	134	0.046
Malignant(III–IV)	49(84.5%)	9(15.5%)	58	
**Histologic type**				
Astrocytoma	105(75.5%)	34(24.5%)	139	0.704
Glioblastoma	26(81.2%)	6(18.8%)	32	
Oligoastrocytoma	13(86.7%)	2(13.3%)	15	
Ependymoma	5(83.3%)	1(16.7%)	6	

*χ^2^ test.

### BRMS1 regulates glioma cells invasion and MMP activity through NF-κB pathway

As cell proliferation and invasion are an important factor for tumor progression and BRMS1 expression is significantly reduced in glioma, we investigated the role of BRMS1 in glioma cells proliferation and invasion. First, we transfected glioma U251 and U87 cells with pFlag-BRMS1 and found that BRMS1 was overexpressed in this cell line compared with control cells (Fig. 2A). Subsequently, 24 hour after transfection, cells were subjected to cell proliferation assay and cell invasion assay. Our data indicated that the cell proliferation rates were similar between control group and the BRMS1 overexpression group in both U251 and U87 cells (Fig. 2B, C). However, in cell invasion assay, BRMS1 overexpression inhibits cell invasive ability of U251 and U87 cells in matrigel-coated Boyden chamber by 42% and 55%, respective (Fig. 2D, E).

**Figure 2:** Overexpression of BRMS1 suppresses cell invasion but not cell proliferation in glioma cells. **A** Twenty-four hours after transfection, the expression of BRMS1 in U251 and U87 glioma cells was evaluated by western blot. **B, C** CCK-8 cell proliferation assay was performed after BRMS1 overexpression in U251 and U87cells. **D, E** Matrigel cell invasion assay was performed after the overexpression of BRMS1 in U251 and U87 cells. The graph shows the percentage of cells invaded in 5 fields of view compared with the control group. **F** BRMS1 inhibits MMP-2 activity in U251 and U87 cells by zymography. **G** Western blot analysis of the relative protein levels of MMP-2, uPA and NF-κB in BRMS1 overexpression and control group of U251 and U87 cells. **H** Quantitative analysis of relative protein level of MMP-2, uPA, p27 and NF-κB in glioma U251 and U87 cells. All experiments were carried out in triplicate. Data are shown as mean ± SD. *P<0.05, **P<0.01.

Since MMPs play a crucial role in cell invasion, we then carried out the zymography assay to compare the activity of MMPs in BRMS1-overexpressing and control cells. As shown in Fig. 2F, MMP-2 gelatinolytic activity was dramatically decreased by 58% and 45% in BRMS1-overexpressing U251 and U87 cells compared with the control cells, respectively. Then, we performed western blot to examine the MMP-2 expression in glioma cells. Western blot results showed that MMP-2 protein level was sharply decreased after BRMS1 overexpressed in U251 and U87 cells (Fig. 2G–H). The urokinase-type plasminogen activator (uPA), being a downstream effector of NF-κB, which is known to activate the MMPs leading to invasion. Our results demonstrated that the NF-κB and uPA expression was dramatically decreased in U251-BRMS1 and U87-BRMS1 cells compared with control cells (Fig. 2G–H).

### BRMS1 inhibits glioma cell migration, adhesion via Src-FAK pathway

Tumor cell adhesion to the extracellular matrix is implicated in tumor cell motility, invasion and metastasis. We then used the migration and adhesion assay to detect if BRMS1 affect cell motility and adhesiveness. First, we investigated the role of BRMS1 in migration of glioma cells by wound-healing assay and migration assay. We found that there was significant delay in wound closure after BRMS1 re-expression compared with pFlag-control transfected group (Fig. 3A, B). In addition, in cell migration assay, our results showed that U251-BRMS1 cells and U87-BRMS1 cells decreased the ability to migrate through Boyden chamber by 62% and 68%, respectively, compared with the control cells (Fig. 3C, D). Moreover, we used the adhesion assay to detect if BRMS1 affects cell attachment ability. We found that cell attachment ability was reduced by 60% and 63% in BRMS1-overexpressing U251 and U87 cells compared with the control cells (Fig. 4A, B).

**Figure 3:** Overexpression of BRMS1 inhibits glioma cell migration. **A, B** Wound-healing assay was done on monolayers of U251and U87 glioma cells after 24 hour of transfection. The photographs were taken at 0 and 24 hours after wounds were made. **C, D** Cell migration assay was performed after overexpression of BRMS1 in glioma U251 and U87 cells. The graph shows the percentage of cells migrated in 5 fields of view compared with the control group. All experiments were carried out in triplicate. Data are shown as mean ± SD. **P<0.01; ***P<0.001.

**Figure 4:** Overexpression of BRMS1 inhibits glioma cells adhesion ability. **A, B** Cell attachment assay after BRMS1 overexpression in U251 and U87 cells. The graph shows the percentage of attached cells compared with the control group. **C** Western blot analysis of the relative protein levels of Src and FAK in BRMS1 overexpression and control group for both U251 and U87 cell lines. **D** Quantitative analysis of relative protein level of Src and FAK in glioma U251 and U87 cells. All experiments were carried out in triplicate. Data are shown as mean ± SD. *P<0.05, **P<0.01.

There is convincing evidence that the activities of Src family kinases and focal adhesion kinase (FAK) control cell migration and adhesion processes and increased expression of these kinases has been associated with more adhesive and aggressive phenotypes [25]–[27]. So we examined the protein levels of Src and FAK by western blot. The Src and FAK expression were significantly suppressed after BRMS1 expression in U251 and U87 cells compared with the control cells (Fig. 4C, D). Our results indicated that BRMS1 might inhibit glioma cell migration, adhesion via Src-FAK pathway.

## Discussion

Metastasis suppressors are a growing family of molecules that are functionally defined by their ability to suppress metastasis without blocking orthotropic, primary tumor growth when re-expressed [28]. BRMS1 gene was originally identified as a true metastasis suppressor gene in breast cancer cell lines as stable overexpression of BRMS1 suppressed pulmonary metastasis. Subsequent studies have indicated that BRMS1 remarkable suppresses the metastatic phenotype in vitro in cells from several other types of cancer, including melanoma, ovarian cancer, bladder cancer, lung cancer [5], [6], [9], [12], [29]. BRMS1 was also shown to inhibit metastasis in xenograft models of these tumors. In addition, BRMS1 has clinical relevance for some tumor types. BRMS1 mRNA expression was downregulated in breast tumor tissues and in breast cancer brain metastases [8], [15]. Zhao et al claimed that BRMS1 expression in ovarian serous adenocarcinoma was significantly lower than in both normal ovarian tissue and benign ovarian tumor tissue [30]. Another study found that BRMS1 expression was diminished in NSCLC compared to the adjacent non-cancerous lung [12]. The relevance of BRMS1 in cancer was reinforced by the identification that BRMS1 downregulation was correlated with poor patient survival in breast cancer, ovarian cancer, melanoma, NSCLC, and nasopharyngeal carcinoma [6], [7], [9], [11], [12]. However, the role of BRMS1 in glioma has not been clearly studied. In this study, our data first demonstrated that BRMS1 is significantly decreased in clinical glioma tissues and glioma cells compared to tumor adjacent normal brain tissue and NHA by Immunohistochemical and Western blot technique (Fig. 1A–G). In addition, BRMS1 expression is downregulated in high grade (III–IV) glioma in comparison to low grade (I–II) glioma (Fig. 1H). The reduced expression of BRMS1 in glioma can possibly be explained by the theory that deletion at chromosome 11q, which includes the BRMS1 gene, occurs at very high frequency in various human cancers [31], [32]. Another study found that the methylation of BRMS1 promoter might account for the loss of BRMS1 in advanced cancer. Our results are consistent with previous findings. This indicated that BRMS1 might play an important role in the glioma development and progression.

Invasion growth is the most characteristic biological phenotype of glioblastoma. In vitro assay, our studies found that overexpression of BRMS1 cannot regulate cell proliferation significantly, but the cell invasion ability is dramatically suppressed in glioma cell lines (Fig. 2B–E). A critical step of invasive tumor cells is the ability to cross the extracellular matrix (ECM) tissue boundaries, a process that can be accomplished by expression of active metalloproteases (MMPs). MMP2 is thought to be key enzymes involved in the degradation of type IV, which is a component of the ECM [33]. High levels of MMP2 in tissues are associated with tumor cell invasion, including glioma [34]. In this study, our data suggested that overexpression of BRMS1 inhibited MMP-2 protein expression and enzyme activity in glioma cell lines (Fig. 2F–H). BRMS1 negatively regulates uPA expression through inhibition of NF-κB activity in breast cancer and melanoma cells [15]. Consistent with those findings, our data showed that overexpression of BRMS1 suppressed NF-κB and uPA expression (Fig. 2G–H). uPA, a serine protease that is known to activate the MMPs leading to invasion [35]. Therefore, our study demonstrated that BRMS1 suppression of glioma cell invasion is mediated via inhibition of NF-κB and subsequent suppression of the uPA and MMP-2.

A multistep model of invasion suggests that cancer cells must first adhere to the ECM, proteolytically degrade the matrix, and finally migrate through this barrier to surrounding tissue [36]. Consequently, it is possible that BRMS1 contributes to glioma tissue invasion by increasing tumor cell migration and adhesion. Indeed, we found that re-expression of BRMS1 decreased cell migration and adhesion abilities of glioma cells (Fig. 3 and 4). Src-FAK signaling cascade have multiple cellular functions and modulation of their activities can alter cellular responses that are often perturbed in cancer cells, such as adhesion, migration, and invasion[37]–[39]. FAK promotes cancer cell migration and adhesion by regulating focal adhesion formation and turnover, which involve activation of Src [40]. Constitutively activated Src-FAK pathway is capable of inducing malignant transformation of a variety of cell types, including glioma [41]. Inhibition of Src-FAK pathway decreased glioma migration and invasion [42]. We found the Src and FAK expression were significantly suppressed after BRMS1 expression in glioma cells. This is suggested that BRMS1 might inhibit glioma cell migration and adhesion through Src-FAK pathway. However, the more exact molecular mechanism of how BRMS1 regulates Src and FAK expression need us further investigation.

In summary, we demonstrated that BRMS1 plays an important role in human glioma pathogenesis. Reduced BRMS1 expression may facilitate tumor progression by enhancing cell invasion, migration and adhesion. Our results imply that targeting of the BRMS1 pathway may constitute a potential treatment modality for glioma.
